RETRACTED

# An Improved COVID-19 Detection using GAN-Based Data Augmentation and Novel QuNet-Based Classification

**DOI:** 10.1155/2022/8925930

**Published:** 2022-02-26

**Authors:** Usman Asghar, Muhammad Arif, Khurram Ejaz, Dragos Vicoveanu, Diana Izdrui, Oana Geman

**Affiliations:** ^1^Department of Computer Science & Information Technology, The University of Lahore, Pakistan; ^2^Electrical Engineering and Computer Science Faculty, Stefan cel Mare University Suceava Romania, Pakistan

## Abstract

COVID-19 is a fatal disease caused by the SARS-CoV-2 virus that has caused around 5.3 Million deaths globally as of December 2021. The detection of this disease is a time taking process that have worsen the situation around the globe, and the disease has been identified as a world pandemic by the WHO. Deep learning-based approaches are being widely used to diagnose the COVID-19 cases, but the limitation of immensity in the publicly available dataset causes the problem of model over-fitting. Modern artificial intelligence-based techniques can be used to increase the dataset to avoid from the over-fitting problem. This research work presents the use of various deep learning models along with the state-of-the-art augmentation methods, namely, classical and generative adversarial network- (GAN-) based data augmentation. Furthermore, four existing deep convolutional networks, namely, DenseNet-121, InceptionV3, Xception, and ResNet101 have been used for the detection of the virus in X-ray images after training on augmented dataset. Additionally, we have also proposed a novel convolutional neural network (QuNet) to improve the COVID-19 detection. The comparative analysis of achieved results reflects that both QuNet and Xception achieved high accuracy with classical augmented dataset, whereas QuNet has also outperformed and delivered 90% detection accuracy with GAN-based augmented dataset.

## 1. Introduction

Corona virus is a respiratory disease caused by the acute respiratory syndrome corona virus 2 (SARS-CoV-2) detected in Wuhan, China, in December 2019. This disease further developed into a global pandemic causing disruption, unemployment, and lockdown all over the world. As of May 2021, 3.8 million people have lost their lives to this disease and 177 million have been affected at the current time. The vaccine existing has not gained confidence at a large scale due to the lack of evidence about its usefulness and possible side effects; therefore, to inhibit further spread, patients need to be tested promptly and isolated for a certain period of time.

The main source of detecting patients affected by COVID-19 remains to be reverse transcription-polymerase chain reaction (RT-PCR) test kits, but despite doctors working day and night at the frontier, detecting COVID-19 is a slow process combined with limited resources in many countries. The result is not always accurate with a lot of false negatives and positives [1]. This virus, however, affects the lungs causing inflammation in air sacs, and as a response, the alveoli to be filled with fluid, which can be detected by examination of X-ray images [2], along with CT scan images and biomarkers.

RETRACTED

As the next wave of corona virus approaches the world in 2021, it has become vital to produce a new methodology for promptly and accurately detecting the disease in patients. So far, several deep learning models have performed significantly in health care for disease classification. However, a catch with deep learning models is that they require a large amount of dataset in order to be trained effectively. A small dataset causes overfitting leading to a lack of generalization, i.e., it picks up noise and details to such a large extent that the model is not able to learn efficiently the features of the disease itself [3]. Since the corona virus is a novel disease, so, the available dataset is limited to train the deep learning models efficiently. Therefore, there is a need to increase the existing dataset to overcome this problem. In this regard, the data augmentation techniques are being opted as a viable option.

The classical data augmentation methods mainly include some techniques such as rotate, scale, zoom, horizontal and vertical on real images and synthetic images generated by generative adversarial network (GAN) as a modern augmentation. A GAN uses two competing parts, generator and discriminator to produce artificial images [4]. This technique can overcome the problem of the limited dataset and improve the accuracy of the deep learning models. In addition, this research work proposes a novel deep learning architecture named as QuNet, which exhibits better performance using GAN-based augmented images. Convolutional neural network (CNN) models, such as InceptionV3, Resnet101, DenseNet-121, and Xception, are trained on augmented dataset using ImageNet weights as well as no preloaded weights to compare the performance of models in terms of accuracy with each other.

The remainder of this research work describes the methodologies of other researchers for the addressed work. Then, proposed methodology is discussed in detail with results and comparative study, and finally, this research work is concluded at the end of this document.

## 2. Related Work

At the peak of this pandemic, a lot of research work [5, 6] has been done as well as in progress to help ease in detecting and treating COVID-19 [7, 8]. With an inclination towards using deep learning models [9, 10] for detection of corona virus, various papers have proposed and showed how to use CNNs and transfer learning to use VGG16, VGG19, ResNet, DenseNet, and other models for fine-tuning and feature extraction in currently available X-ray and CT scan dataset.

RETRACTED

Waheed et al. [1] presented a method for generating chest X-ray images by using auxiliary classifier generative adversarial network- (ACGAN-) based model called CovidGAN. Data augmentation for dataset extension was employed. Furthermore, these images were used to show that using synthetic images can improve the accuracy of CNN in COVID-19 detection. Thapa and Camtepe [11] proposed a deep learning-based technique for the detection of COVID19 using the radiological image dataset. Their approach comprised of a twofold classification of raw chest X-ray images as binary classification and multiclass classification. The prominent part of the study is that it performed the classification without utilizing the feature extraction technique; instead, it focused on the proposed dark classifier. Moreover, the model used the Cohen JP dataset of 127 X-ray images of COVID-19 positive patients, and it was trained and tested using two other classes, namely, pneumonic and healthy, comprising of 500 images each. Additionally, the state-of-the-art YOLO architecture in combination with a dark classifier was used in this study for archiving optimal results. Additionally, the lack of the image dataset also caused ambiguity among the researchers themselves.

Similarly, Nayak et al. [12] proposed the use of transfer learning for deep CNN architectures. The study is aimed at performing robust detection of COVID-19 cases by using a deep learning and convolutional neural network-assisted model. Meanwhile, the early detection of the COVID-19 was carried out by validating the model on two different X-ray image datasets that are covidchest-x-ray-dataset and ChestXray8. These datasets comprised 203 frontal chest X-ray images of COVID-19 positive patients. Along with that, the study used two classes as health and COVID-19 for effective training and classification of the deep CNN model. Additionally, the study effectively eliminated the imbalance and scarcity factor of available data by performing offline data augmentation of scare image datasets. Eight state-of-the-art deep CNN models, namely, ResNet-50, AlexNet, SqueezeNet, Inception-V3, GoogleNet, VGG-16, MobileNet-V2, and ResNet-34, were used for the comparison of the effectiveness of the proposed method. The ResNet-34 achieved the highest results with 98.33% accuracy that was comparable with [13, 14]. However, the model is not fully reliable as these results are validated on extensively smaller datasets, and multiclass classification can be included in the study for increasing the authenticity and reliability of the published work.

RETRACTED

Mangal et al. [15] suggested a similar technique of performing automated detection of COVID-19. The study comprised of using a deep neural network model for the detection of the deadly disease known as COVID-19 by using radiographic scan images. The authors have presented CovidAID a deep learning and CNN-assisted system that automatically recommends potential patients for actual COVID-19 testing. Therefore, the research aimed to not detect the virus itself but the likeliness of the presence of the virus. Moreover, similar to prior attempts, the proposed system is also trained using the radiographic X-ray scan images of the frontal chest side. The proposed system was trained using 115 corona positive X-ray images along with 1341 normal and about 3000 pneumonic images. Moreover, the state-of-the-art benchmarked system COVID-Net was used for comparing the performance of the proposed system. According to the published document, the system achieved an accuracy of 90.05%; however, it can be seen that the system suffered from the imbalanced distribution of the classification dataset that has affected the results. The proposed system shall need to be validated on a larger dataset to eliminate any remaining concerns of overfitting. Ahuja et al. [16] explored a similar area while considering the computed tomographic images instead of X-ray images. The authors proposed a novel three-phase deep learning technique using wavelets for the detection of COVID-19 from the CT images. The initial proposed phase consisted of performing data augmentation by normalizing and changing the input, size, and type of the images. The middle stage involved utilizing pretrained state-of-the-art CNN models for performing the detection by using the images. Moreover, the final phase addressed the localization of abnormality factors in the used dataset. SqueezeNet, ResNet18, ResNet101, and ResNet50 are state-of-the-art CNN models used for the evaluation of the proposed system. Additionally, the proposed system was validated using a novel dataset comprising of 349 and 397 CT images of COVID-19 and healthy patients, respectively. The 70% and 30% data from the dataset were used for training and testing the proposed system, respectively. However, 99.82% accuracy was delivered by the ResNet18 model that is the result of the overfitting. Even though the authors emphasized the data augmentation, they were unable to present a benchmarked solution that addressed the overfitting dilemma.

RETRACTED

Karakanis et al. [17] introduced a novel deep CNN architecture to facilitate the detection process. In this study, the authors have presented a novel methodology of using general adversarial networks to address the overfitting problems caused by the scarcity of data. Additionally, the authors have made another contribution by presenting two novel lightweight CNN architectures for binary and multiclass classification of input images. Moreover, a previously presented testing protocol was used to evaluate the performance of the proposed architectures. Along with that, the proposed architectures were trained using state-of-the-art transfer learning-based CNN models, and validation was performed by using two different datasets, namely, GitHub-covid-X-ray and Cohen JP. The cGAN was used to generate about 130 synthetic images making the overall total as 275 COVID-19 radiographic, 275 pneumonic, and 270 normal images. However, while the proposed system for binary classification delivered an accuracy of 98.7% along with ResNet8, the system by far is still limited due to the limitation of the data. Though the proposed system has been proven robust and effective in comparison with existing benchmarked solutions, they still need to be validated using a comparatively larger dataset. Wu et al. [18] adopted a similar approach for the classification of COVID-19 using computed tomography images. However, the novel part of the study can be expressed as the usage of classical and conditional GAN augmentation that enlarged the limited dataset. The study used the COVID-19 CT image dataset from GitHub comprising of 742 computed tomography images of two types, namely, COVID-19 and non-COVID-19. However, similar to previous studies the authors also utilized the deep learning-based transfer learning-assisted state-of-the-art CNN models including VGG19, GoogleNet, AlexNet, ResNet50, and VGG16. Additionally, the use of the proposed methodology can be described as the biggest contribution of the study that would significantly enlarge the dataset, and hence, results would be improved. However, the classical data augmentation assisted with deep transfer learning delivered the best accuracy of 82.91% which was comparable with [19, 20]. Moreover, while there were concerns about a benchmark data augmentation [21], the authors also emphasized testing the accuracy on a nonsynthetic images dataset to effectively diagnose the deadly disease.

## 3. Proposed Methodology

Our addressed research work is twofold: the first part consists of data augmentation using classical and GAN-based techniques. In the second part, we have employed the transfer learning using convolutional neural network models including InceptionV3, Resnet101, DenseNet-121, and Xception along with a novel convolutional neural network architecture that has been designed and implemented for the addressed problem and named it the QuNet. The flow diagram of proposed research work is shown in Figure 1.

RETRACTED

### 3.1. Dataset

The CORD-19 open research dataset is used in this research work, and the sample images are shown in Figure 2. In the dataset, three classes are used for training and testing like as COVID-19, pneumonia, and normal. Dataset is cleaned to use only confirmed cases and we normalized the images in data augmentation because of variation in their size.

### 3.2. Classical Augmentation

We used classical data augmentation techniques in image preprocessing for introducing variety in the dataset, to reduce the overfitting and improve the performance of the models. We have applied various classical data augmentation functions including zoom, horizontal shift, vertical shift, and rotation on the dataset to introduce variance.

### 3.3. GAN-Based Augmentation

Additionally, GANs are also used to generate images for each class and the statistics are shown in Table 1 after the classical and GAN-based data augmentation. The GAN architecture has two neural networks, and we trained them together. One neural network is called a generator which takes random noise vector as an input and focuses on generating images; meanwhile, the other neural network, called discriminator, focuses on distinguishing between real and fake images. The architecture of GAN used for data augmentation in our proposed work is shown in Figure 3.

Dataset is further divided into training set, validation set, and test set for the training and evaluation of the proposed and competitive technique. The models are trained with and without GAN-based augmentation. The division of the data is shown in Table 2. The dataset contains images of different sizes which are all later normalized to the size of 224 x 224 each to make the computation efficient.

### 3.4. Loss Graph for GAN-Based Augmentation

Graph in Figure 4 shows the loss details for COVID-19 image dataset output with almost constant loss in discriminator and a high decrease in the generator at the start and similar fashion of decrease at the end.  Figure 5 shows results for the pneumonia class, whereas graph Figure 6 shows the results for the normal class of images generated.

### 3.5. Proposed Deep Learning-Based Classification

QuNet is a novel convolutional neural network that we have designed and used in this research work. The architecture is based on convolutional and MaxPooling layers and uses ReLu as an activation function in Conv2D layers. A dropout layer is used to hinder all neurons from converging to the same goal to prevent overfitting. The MaxPooling layer utilized filters of size 2 × 2, whereas Conv2D layers used filters of size 3 × 3. The first layer of Conv2D takes input of shape 224 × 224 × 3, with ReLu activation function and 1792 parameters. After this layer, another Conv2D layer is applied followed by a MaxPooling2D layer.

RETRACTED

In this sequence, a set of Conv2D layers is used followed by the MaxPooling2D layer and another set with the same parameters. Lastly, two Conv2D layers are followed by one MaxPooling2D layer. Flatten layer follows the sequence, ending the network with a dense, dropout, and dense layer. A total of 268,547 trainable parameters are used. The architecture of the model is shown in Figure 7.

### 3.6. Transfer Learning Using Existing Architectures

In addition, we employed transfer learning technique for training InceptionV3 [22], Xception [23], ResNet [24], and DenseNet-121 [25] models. The transfer learning is applied in two ways: (1) using weights of existing models trained on X-ray images and (2) using weights of models trained on ImageNet dataset.

All these models use convolutional neural networks for training the models. Same architectures are used to train the model and identify COVID-19, pneumonia, and normal images. These convolutional layers extract the features from the images by using filters. Multiple filters can be used to extract the different types of features, whereas the MaxPooling layer passes a filter over each image to extracts the maximum value from all the values in the filter. The main function of this is to reduce image dimension. Each of these filters in convolution computed a dot product with pixel values over a small region over an image producing a feature map.

For image I, the size of filter L is given by Equation (1):

(1) $$\begin{array}{c} \left(I*L\right)r,s=\overset{h1}{\underset{u=-h1}{\sum }}\overset{h2}{\underset{u=-h2}{\sum }}K_{u,v}l_{r+u,s+v}. \end{array}$$

We perform transfer learning as a predictive modeling problem that uses image data as input for training, while some weights of some layers can be kept frozen or unchanged. For computer vision tasks, many models are available for transfer learning including ResNet, DenseNet, Inception, and Xception. The architecture of DenseNet-121 model is used except the fully connected layers which are replaced by our layers. The weights are trained on our dataset as well as ImageNet weights. The whole architecture of InceptionV3 is used to make use of label-smoothing, factorized 7 × 7 convolutions, and the use of an auxiliary classifier to propagate label information lowers down the network. Accuracy is better with ImageNet weights. Xception is a convolutional neural network with deep architecture of 71 layers and it relies on depth wise separable layers. Xception produces 90% accuracy with ImageNet weights. The ResNet-101 mostly used as backbone architecture and it builds on constructs known from pyramidal cells in the cerebral cortex.

RETRACTED

## 4. Results and Discussion

To compare the result, different evaluation metrics are used including precision, recall, and accuracy. All of these evaluation metrics are used extensively in the domain of deep learning for healthcare. The proposed system is evaluated using the following metrics:

### 4.1. Experimental Metrics

Precision is the proportion of positive disease predictions that have actually the said disease. It is calculated using Equation (2):

(2) $$\begin{array}{c} Precision=\frac{Correctly\;classified\;positive\;images}{Total\;classified\;positive\;images}. \end{array}$$

Recall is the ability of proposed model to detect all the potentially diseased images. It is calculated as Equation (3):

(3) $$\begin{array}{c} Recall=\frac{Correctly\;classified\;positive\;images}{Total\;classified\;positive\;images\;\text{in }dataset\;}. \end{array}$$

Accuracy is the measure of correct classification of infectious disease by the proposed system and it is defined as Equation (4):

(4) $$\begin{array}{c} Accuracy=\frac{TP+TN}{Total\;sample\;\text{in }dataset} \end{array}$$

### 4.2. Training Accuracy and Loss Graphs

The following graphs in Figures 8 and 9 are showing the accuracy and loss for the novel QuNet model using the GAN-based augmented dataset and without the ImageNet weights.

After training the models, the following Table 3 and Figure 10 show the results of different models with the classical augmented dataset. Furthermore, results with no preloaded weights and ImageNet weights are shown as well.

Results are shown in terms of accuracy and recall.

Overall QuNet gives the most accurate results in terms of accuracy among all five models. With preloaded weights, QuNet gives 92.92% accuracy followed by

DenseNet-121 and Xception.  Figure 11 shows the confusion matrix for QuNet which is tested with 105 images for each class and label 0, 1, and 2 representing the class COVID-19, pneumonia, and normal. The accuracy obtained is 92%. With ImageNet weights, the DenseNet-121 has the highest accuracy among the four models, whereas ResNet101 gives the least accuracy in all cases.

Table 4 and Figure 12 shows the results for GAN bases data augmented images. QuNet again gives the highest accuracy among all models, whereas ResNet101 shows the least accuracy. DenseNet-121 gives 86% accuracy with no preloaded weights followed by InceptionV3 and Xception. The DenseNet-121, InceptionV3, and Xception provide almost the same accuracy with preloaded weights.

RETRACTED

## 5. Conclusion

The COVID-19 has been designated as a world pandemic by the World Health Organization, and as the infection rate is increasing rapidly around the globe, there is a need for a robust disease detection mechanism. In this study, we have employed the use of various deep learning-assisted CNN models to detect and classify the COVID-19-infected patients using radiographic images such as X-ray images. Furthermore, to overcome the data scarcity problem, we have experimented with the use of augmentation techniques, namely, classical data augmentation and GAN-based data augmentation. Additionally, we have also proposed a novel CNN model QuNet for the improved detection of the virus from the radiographic images. The QuNet model used here is a novel architecture with multiple convolutional layers. It shows promising results in the detection of COVID-19 by using X-ray images. Moreover, GAN-based augmentation also assisted greatly to increase the dataset by generating synthetic X-ray images for the classes of COVID-19, pneumonia, and normal class to solve the problem of overfitting. We also experimented with the research by using the CNN models with ImageNet weights and without any preloaded weights. The approach allowed us to examine the performance of different models under different situations. However, the comparative results indicate that the proposed QuNet delivered a high accuracy of 92% and 90% using classical and GAN-based augmented datasets, respectively, and these results are achieved without using the pretrained ImageNet weights. The results of our trained model are encouraging and graph-charts showing the maturity of our proposed novel QuNet architecture. Meanwhile, the proposed study does not outline the perfect automated system for the detection of the novel COVID-19; however, the model can be validated on larger datasets to validate the real case implementation of our methodology.

## Figures and Tables

**Figure 1:** Proposed work flow diagram.

**Figure 2:** (a) COVID-19 X-ray image sample. (b) Pneumonia X-ray image sample. (c) Normal X-ray image sample.

**Figure 3:** Architecture of generative adversarial network for data augmentation.

**Figure 4:** Loss generating COVID-19 images.

**Figure 5:** Loss generating pneumonia images.

**Figure 6:** Loss generating normal images.

**Figure 7:** Proposed model complete architecture.

**Figure 8:** QuNet accuracy using GAN-based augmented dataset.

**Figure 9:** QuNet loss using GAN-based augmented datasets.

RETRACTED

**Figure 10:** Results with classical augmented dataset.

**Figure 11:** Confusion matrix for QuNet model with GAN-based data augmentation. Label 0 = COVID − 19, Label 1 = pneumonia, and Label 2 = normal.

**Figure 12:** Results with GAN-based augmented dataset.

**Table 1:** Dataset statistics after classical and GAN-based data augmentation.

Class name	Images after augmentation		
	Original	Classical Data augmentation	GAN-based data augmentation
COVID-19	150	560	710
Pneumonia	150	560	710
Normal	150	560	710

**Table 2:** Dataset split after classical and GAN-based augmentation.

Augmentation method	Class	Training images	Validation images	Test images
Classical	COVID-19	400	80	80
	Pneumonia	400	80	80
	Normal	400	80	80

GAN-based	COVID-19	500	105	105
	Pneumonia	500	105	105
	Normal	500	105	105

**Table 3:** Results with classical augmented dataset.

Model	No weight		ImageNet weight	
	Accuracy	Recall	Accuracy	Recall
DenseNet-121	0.8500	0.900	0.9125	0.7500
Inception V3	0.6500	0.8875	0.8417	0.7250
Xception	0.7375	0.8375	0.9208	0.7875
ResNet101	0.6625	0.0125	0.6542	0.9625
QuNet	0.9292	0.8250	————–	———-

**Table 4:** Results with GAN based augmented dataset.

Model	No weight		ImageNet weight	
	Accuracy	Recall	Accuracy	Recall
DenseNet-121	0.8635	0.6667	0.8730	0.7333
Inception V3	0.7556	0.8667	0.8508	0.8095
Xception	0.7683	0.6857	0.8571	0.6857
ResNet101	0.6540	0.8571	0.3333	1.000
QuNet	0.9000	0.7714	————–	———-

## Data Availability

The data used to support the findings of this study are available from the corresponding author upon request.
